# Databases and Bioinformatics Tools for the Study of DNA Repair

**DOI:** 10.4061/2011/475718

**Published:** 2011-07-14

**Authors:** Kaja Milanowska, Kristian Rother, Janusz M. Bujnicki

**Affiliations:** ^1^Laboratory of Bioinformatics and Protein Engineering, International Institute of Molecular and Cell Biology, ul. Ks. Trojdena 4, 02-109 Warsaw, Poland; ^2^Laboratory of Bioinformatics, Institute of Molecular Biology and Biotechnology, Adam Mickiewicz University, ul. Umultowska 89, 61-614 Poznan, Poland

## Abstract

DNA is continuously exposed to many different damaging agents such as environmental chemicals, UV light, ionizing radiation, and reactive cellular metabolites. DNA lesions can result in different phenotypical consequences ranging from a number of diseases, including cancer, to cellular malfunction, cell death, or aging. To counteract the deleterious effects of DNA damage, cells have developed various repair systems, including biochemical pathways responsible for the removal of single-strand lesions such as base excision repair (BER) and nucleotide excision repair (NER) or specialized polymerases temporarily taking over lesion-arrested DNA polymerases during the S phase in translesion synthesis (TLS). There are also other mechanisms of DNA repair such as homologous recombination repair (HRR), nonhomologous end-joining repair (NHEJ), or DNA damage response system (DDR). This paper reviews bioinformatics resources specialized in disseminating information about DNA repair pathways, proteins involved in repair mechanisms, damaging agents, and DNA lesions.

## 1. Introduction

DNA repair processes are indispensable for maintaining the integrity of genetic information in all organisms. Environmental agents such as chemicals, UV light, and ionizing radiation, as well as endogenous metabolic processes involving DNA constantly challenge the chemical structure and stability of the genome. DNA lesions can interfere with processes such as DNA replication or transcription and may lead to mutations and cancer [1, 2]. To prevent the erosion of the chemical structure of DNA, living systems have evolved various different biochemical systems for DNA repair [3–7]. 

DNA damage from endogenous sources gives rise to 20,000 lesions per mammalian cell per day. Amongst these lesions, the most common are base deamination, spontaneous hydrolysis of the *N*-glycosidic bond, alkylation, and damage by reactive oxygen or nitrogen species and lipid peroxidation products [8–12]. Other lesions such as the formation of single- and double-strand breaks, the collapse of replication forks, and the introduction of modified nucleic acid bases during DNA replication are caused by errors in DNA metabolic processes. In total, there are 10^16^–10^18^ DNA repair events that occur daily in a healthy adult man (10^12^ cells) [13]. Lesions that are not repaired often lead to mutations, aging and various diseases, including carcinogenesis and neurodegeneration [14–18]. Some pathological disorders directly related to defects in the DNA repair machinery are Xeroderma pigmentosum, different types of cancer (breast cancer, colorectal cancer, endometrial cancer, gastric cancer, or prostate cancer), Fancomi anemia, Muir-Torre syndrome, Tay syndrome, and Werner syndrome. On the other hand, unrepaired lesions that occur in germline cells become the main source of genetic variability and therefore a driving force for the evolution. For this reason, the DNA repair system needs not only to be regulated to maintain an individual genome's integrity, but also to increase the genetic variability in the context of populations. Many mechanisms are known that regulate the amount of DNA repair as a response to environmental conditions [19].

Given its many duties in different contexts, it is not surprising that DNA repair is a very complicated process, involving many factors. For instance to date, 168 genes encoding proteins involved in DNA repair have been identified in the human genome [17, 18, 20] (20 January 2011, date last accessed). Over all organisms, there are many more; for base excision repair alone, KEGG [21] lists 41 groups of orthologous genes encoding for hundreds of proteins in total. The key players in DNA repair are enzymes that catalyze reactions leading from the DNA with damage to a repaired molecule. They are assisted by proteins that detect damage and mediate signals that coordinate the repair process with other cellular processes. From the point of view of the DNA substrate, the biochemical pathways of DNA repair can be divided into eight categories:

- DNA damage signaling (DDS): also known as the DNA damage checkpoint; it is a group of responses to DNA damage caused by some endogenous and environmental agents; activation of these pathways may be triggered by the effect the DNA lesions have on replication, transcription, or chromatin topology;
- base-excision repair (BER): initiated by excision of a modified base from the DNA. Depending on the length of DNA resynthesis, the pathway is subdivided into two subpathways: short path (SP-BER) or long path (LP-BER);
- DNA damage response (DDR): directly restores the native nucleotide residue by removing the nonnative chemical modification;
- homologous recombination repair (HRR): repair of DNA double-strand breaks using the homologous DNA strand as a template for resynthesis;
- mismatch repair (MMR): postreplicational DNA repair that removes errors introduced during the replication (misinserted nucleotides, small loops, insertions, deletions);
- nonhomologous end-joining repair (NHEJ): ligation of ends resulting from DNA double-strand breaks (including the more error-prone microhomology-mediated end-joining (MMEJ) mechanism;
- nucleotide excision repair (NER): removes bulky damage from the DNA. The damage from the active strand of transcribed genes is removed by transcription coupled repair (TCR)-NER, while global genome repair (GGR)-NER removes damage present elsewhere in the genome;
- translesion synthesis (TLS): damage-tolerance pathway that employs specialized polymerases to replicate across lesions in order to finish replication despite DNA damage.

Each of these pathways can be represented as a series of enzymatic transformations between different DNA structures, catalyzed by a dedicated system of proteins. It must be emphasized that DNA repair pathways are connected to each other, that is, they can share some steps and/or proteins involved [13]. As a consequence, DNA repair proteins rarely work in isolation in the cell, and their activity is dependent on other components of DNA repair systems. 

DNA repair itself is not an isolated process, and it is strongly connected to other pathways of nucleic acid metabolism, including (but not limited to) DNA replication, DNA epigenetic modification, transcription, cell cycle regulation, and induced cell death as well as processes that are specific to different domains of life, such as telomere maintenance in eukaryotes and DNA restriction in prokaryotes.

## 2. DNA Repair Data and Databases 

The knowledge of DNA repair systems and their components is critical to our understanding of how cells control the integrity of their genomes. A large body of data on this topic has been published mostly in the literature and in a few electronic resources. Today, systematizing this knowledge and presenting it in a clear and easily accessible way is mostly done by biological databases. The collection, curation, and availability of data are necessary to answer questions about subsystems of DNA repair, for example, “which proteins participate in MMR in humans and in plants?”, “what immediate cellular response is triggered by damage caused by UV light?”, or “how does HRR differ between plants and vertebrates?”. The topic of DNA repair is covered by many computational resources. However, there are few databases dedicated to DNA repair, and most of the data is scattered over various general databases. In Table 1, we have listed some of the available web resources relevant to DNA repair, and in the following section we discuss their content.

### 2.1. Databases Dedicated to DNA Repair

“REPAIRtoire” is a database for systems biology of DNA damage and repair developed by the authors of this paper and their coworkers [22]. The purpose of this database is to gather information about all DNA repair systems and proteins from model organisms and to facilitate the access to knowledge about correlation of human diseases with mutations in genes responsible for DNA integrity and stability as well as information about toxic and mutagenic agents causing DNA damage. REPAIRtoire is available online at http://repairtoire.genesilico.pl/. It organizes data into the following categories: (i) the chemical structures of DNA lesions (as of April 2011: 85 different types of damage in the DNA) linked to their causative mutagenic and cytotoxic agents, (ii) pathways comprising individual processes and enzymatic reactions involved in the removal of damage, (iii) proteins participating in DNA repair, in particular enzymes involved in the transformation between different chemical structures of the DNA substrate, and (iv) diseases correlated with mutations in genes encoding DNA repair proteins (40 diseases caused by the mutations in 32 genes linked to defects in DNA repair proteins). It also provides links to publications and external datasets. REPAIRtoire covers all eight main DNA damage checkpoint, repair, and tolerance pathways (see above). The pathway/protein dataset is currently limited to three model organisms: *Escherichia coli*, *Saccharomyces cerevisiae*, and *Homo sapiens*. DNA repair and tolerance pathways are represented as graphs and in tabular form with descriptions of each repair step as well as corresponding proteins. The individual entries in the database (proteins, diseases, pathway steps, damage, etc.) are cross-referenced to the supporting literature and their respective primary databases. REPAIRtoire can be queried by the names of pathway, protein, enzymatic complex, damage and disease. The query tool returns a structured list of entries in the database that contain the query (e.g., “cancer”, “DNA polymerase”, “crosslink”, “adenine”, etc., or a name of the author). 

The REPAIRtoire website provides a system for editing, adding, and removing data. These features have been provided for collaborators and “superusers” who are interested not only in viewing, but also curating the content of the database. Creating an account and logging into the database grants access to the administrative site of the database to a user. By entering the administration site, it is possible to add new data, delete information, edit, and correct mistakes. Editing information about proteins, genes, diseases, and types of damage is also available via wiki-like pages for particular database entries. Users can also add comments and suggest new references for the existing records. REPAIRtoire is unique in that it focuses on DNA repair and provides reciprocal annotation between damage entities and the proteins that can detect and remove them. It also contains more connections between DNA lesions and the respective proteins that can detect and remove them than can be found in general-purpose databases.

The REPAIRtoire website which also provides an online tool for drawing images of DNA-protein complexes (accessible via the “draw a picture” link in the main menu) is provided. This tool has been developed to illustrate all steps of DNA repair pathways as protein-DNA complexes, in which proteins are displayed in the textbook-like format of “potato models” (ellipsoids). However, it can be also used outside the DNA repair context to create images of any protein-protein or protein-DNA complexes. The drawing engine uses the SVG format provided by the W3C consortium and enables exporting the image in the JPEG format. Images created in the SVG vector format can be scaled without losing quality and can be modified with external tools for vector graphics processing, for example, Inkscape or other free or commercially available software.

The “*repairGENES*” database (http://www.repairgenes.org/) collects information about genes encoding proteins involved in DNA repair and connects information taken from sequence and ontology databases. At the moment, the site contains DNA repair genes from 134 selected species. The database can be browsed by organisms and by biological processes defined by the Gene Ontology (GO) standard [42]. The species are organized in a taxonomy tree. For processes, 17 subcategories of the GO term “DNA repair” (GO:0006281) and their respective subterms are distinguished. For each process, the organisms and genes that refer to this term can be listed. Also, it is possible to highlight the processes for a given organism. The major advantage of using GO terms is that they are being used ubiquitously for annotating sequence data. The raw data about DNA repair genes is extracted from the SWISS-PROT database. The repairGenes database also gives an overview of DNA repair processes and genes in five selected organisms (*Archaeoglobus fulgidus*, *Drosophila melanogaster*, *E. coli*, *Homo sapiens*, and *S. cerevisiae*), in total listing 452 genes. 

“*Human DNA Repair Genes*” is an online supplement to a review published by Wood et al. in 2005 [17] and updated regularly (http://sciencepark.mdanderson.org/labs/wood/DNA_Repair_Genes.html). It provides a table with Gene Name (synonyms) linked to the GeneCards Human Gene Database at Cancer Research UK (http://bioinformatics.cancerresearchuk.org/genecards/) [43], activity linked to the OMIM database, chromosome location linked to the NCBI MapView, and an accession number linked to the NCBI Entrez server [44]. 

The “*Repair-FunMap*” database [23] used to provide information about the network of interactions between proteins involved in DNA repair and other proteins, but to our best knowledge it is no longer available.

### 2.2. General-Purpose Databases Relevant to DNA Repair

“*KEGG*” (Kyoto Encyclopedia of Genes and Genomes, available at http://www.genome.jp/kegg/) [21] is a collection of separate cross-linked databases including KEGG PATHWAY, KEGG DISEASE (human diseases), KEGG GENES (genes and proteins), and KEGG ORGANISMS. Of particular relevance to DNA repair are KEGG GENES (a catalog of genes for sequenced genomes obtained from publicly available resources, mostly NCBI RefSeq and KEGG PATHWAY (a collection of manually drawn pathway maps representing knowledge on the molecular interaction and reaction networks for: global map of pathways, metabolism, genetic information processing, environmental information processing, cellular processes, organismal systems, human diseases, and interaction of these systems with drugs)). DNA repair pathways annotated in KEGG include BER, NER, NHEJ, MMR, and HRR but not DDS, DDR, or TLS. A schematic graphical representation of protein-DNA complexes in the reaction steps of each pathway is available for Eukaryotes and Prokaryotes separately. KEGG BRITE is another component of KEGG that is important for analyzing DNA repair systems. It is a collection of hierarchical classifications representing knowledge on various aspects of biological systems. In contrast to KEGG PATHWAY, which is limited to molecular interactions and reactions, KEGG BRITE incorporates many different types of relationships. The most relevant and interesting part is a section devoted to DNA repair (identifier “ko03400”—“DNA repair and recombination proteins”), where all DNA repair proteins available in KEGG are classified according to their functions in this process.

“*Reactome*” (http://www.reactome.org/ReactomeGWT/entrypoint.html) [24] is a resource developed in collaboration among different groups as an open source curated bioinformatics database of human pathways and reactions. The site provides bioinformatics tools for pathway analysis such as: the Pathway Browser, the Pathway and Expression Analysis tools, or the Species Comparison tool. In contrast to KEGG, Reactome includes graphical representations of DNA repair pathways generated for each organism explicitly instead of a generalized view like in KEGG. Moreover, Reactome divides pathways into subpathways, for example, GG-NER (global genomic NER) in human is divided into four subpathways (DNA damage recognition, formation of the incision complex, dual incision reaction, and gap-filling DNA repair synthesis and ligation). Each subpathway contains individual reactions visualized in the context of the entire cellular metabolic map. The Pathway Analysis tool facilitates analysis of different pathways, for example, finding connections between RNA transcription and DNA repair, facilitating interdisciplinary studies [45].

The “*GeneSNPs*” database (http://www.genome.utah.edu/genesnps/) is dedicated to known human polymorphisms and has a section devoted to DNA repair. It can be accessed from the main page by selecting “DNA repair” in the Gene Lists menu on top of the home page. The SNP loci are presented as a table of 119 human genes involved in DNA repair and connected to phenotypes described in the OMIM database [44]. An exemplary usage of this resource is the study of polymorphisms in the DNA repair gene XRCC, where all the SNP data were collected from the GeneSNPs database [46]. More phenotypes of DNA repair defects can be found in the “*Mouse Mutation Database*” (a database of mouse strains carrying targeted mutations in genes affecting cellular responses to DNA damage available at http://pathcuric1.swmed.edu/research/research.htm) [25].

“*BioCyc*” (http://biocyc.org/) [26] is a collection of 1004 (as of February 2011) Pathway/Genome Databases. Each database in the BioCyc collection describes the genome and metabolic pathways of a single organism. This is not only a collection of databases but of tools for bioinformatics analysis, including the following: a genome browser, a display of individual metabolic pathways and of full metabolic maps, visual analysis of user-supplied “omics” datasets by painting onto metabolic, regulatory, and genome maps, and comparative analysis tools. There is also downloadable version of BioCyc that includes the Pathway Tools. The BioCyc databases are divided into three tiers, based on their quality. Tier 1 databases have received person-decades of literature-based curation and are the most accurate. These include for example, EcoCyc (http://ecocyc.org/) [47], a comprehensive database of *Escherichia coli* K-12 MG1655 biology or MetaCyc (http://metacyc.org/), a database of nonredundant, experimentally elucidated metabolic pathways. Data included in these databases undergo a curation procedure involving external experts, who work on particular cellular systems to provide a comprehensive literature overview and up-to-date coverage of the field. Recently, this type of curation has been applied to the process of DNA repair; both direct repair mechanisms, such as photolyase, as well as indirect repair mechanisms, such as nucleotide excision repair, base excision repair and homologous recombination have been annotated [47]. Tier 2 and Tier 3 databases of BioCyc contain computationally predicted metabolic pathways, predictions as to which genes code for missing enzymes in metabolic pathways, and predicted operons. BioCyc does not include a dedicated DNA repair section, but information on DNA repair pathways can be found in other database sections. Data available in BioCyc can be used in in-depth analyses of biological systems relevant to different fields of research. This approach has been demonstrated in the study of differential network expression during drug and stress response by Cabusora et al. [48], where the expression data of known stress responders and DNA repair genes in mycobacterium tuberculosis from BioCyc collection were used.

“*BRENDA*” (BRaunschweig ENzyme Database, http://www.brenda-enzymes.org/) [27] is a comprehensive database on enzymes that collects manually annotated information on properties of enzymes, including mutants and engineered variants. It describes enzymes involved in DNA repair that have an E.C. number (e.g., uvrA: EC 3.1.25.1). Enzyme records contain data taken from the primary literature, such as classification, nomenclature, reaction type, substrate specificity, functional parameters, species, protein sequence and structure, practical application, information on mutants and engineered variants, stability, disease, isolation, and preparation. An essential part of BRENDA consists of information on metabolites and small molecules, which interact with enzymes as substrates and products, inhibitors, activating compounds, cofactors, or bound metals. BRENDA provides also enzyme disease-related information obtained from PubMed entries by text-mining procedures. BRENDA is currently the largest continuously maintained and publicly available enzyme database and covers a large number of experimentally characterized DNA repair enzymes.

“*Pathway Commons*” (http://www.pathwaycommons.org/pc/) is a comprehensive collection of publicly available pathway data from multiple organisms [28], which includes biochemical reactions, complex assembly, transport, catalysis events, and physical interactions involving proteins, DNA, RNA, small molecules, and complexes. This meta-database collects information from other databases such as Reactome or BioGrid, thereby facilitating analyses of system-level datasets across several species. It allows users to browse and search pathways across multiple valuable public pathway databases and download an integrated set of pathways in the BioPAX format for global analysis. It also provides an interface for software developers to create software for more advanced analyses and hence may be a very useful resource for programmatic linking of data on DNA repair systems with other cellular systems and pathways. 

There exist numerous databases dedicated to other aspects of DNA metabolism. Examples include DNA replication (OriDB [34], ReplicationDomain [41]), apoptosis (Deathbase [49]), telomere maintenance (Telomerase database [40]), DNA restriction and modification (REBASE [35]), and epigenetics/chromatin modification (DAnCER [39]). These processes are relevant to DNA repair as they may contribute to DNA damage (replication) or regulation of other enzymatic processes (DNA methylation, cell cycle control, and apoptosis).

## 3. Bioinformatics Tools for the Study of DNA Repair Proteins

In addition to databases that store and disseminate the data, there are also bioinformatics tools that can be particularly useful for data analyses. We would like to emphasize three groups of predictive tools that can be particularly useful for analyzing DNA repair enzymes: methods for predicting and modeling protein structures, predicting protein-DNA interactions and complexes, predicting the effect of amino acid substitutions on protein stability and function, and their phenotypic effect [50], as well as predicting cancer outcome [39]. 

### 3.1. Protein Structure Prediction

There is a large number of tools, with which to predict the structure of a protein when only its sequence is known. Their performance is evaluated in the biannual CASP benchmarking experiment [51]. One approach we would like to highlight here is homology modeling. There, a protein with known 3D structure is used as a template to construct a model for another, evolutionarily-related protein (a target). This approach requires not only an experimentally solved structure of the template protein, but also a pairwise sequence alignment between the target and the template. Among the numerous methods, the “*SWISS-MODEL*” server (http://swissmodel.expasy.org/) supports not only the fully automatic construction of homology models via its web interface, it also helps finding a suitable template and alignment [52]. It is particularly useful for building models of proteins that are closely related to the experimentally determined structures, so the relationship can be detected by methods such as “*BLAST*” [53]. If no such closely related templates are available, advanced template search and alignment tools such as “*HHSEARCH*” [54] can be used to identify remote evolutionary relationships. There are also specialized “meta-servers” such as the “*GeneSilico Metaserver*” [55] developed in the laboratory of the authors of this paper. These tools use several third-party methods and infer a consensus prediction.

As an example of protein modeling application to the analysis of DNA repair, we may refer to an analysis carried out in our laboratory: Missense alterations of the mismatch repair gene MLH1 have been identified in a significant proportion of individuals suspected of having Lynch syndrome, a hereditary syndrome that predisposes for cancer of colon and endometrium. The pathogenicity of many of these alterations was, however, unclear. A number of MLH1 alterations are located in the C-terminal domain (CTD) of MLH1, which is responsible for constitutive dimerization with another protein PMS2. We used the aforementioned “*GeneSilico Metaserver*” [55] to identified structurally characterized homologs of MLH1 and align their sequences, thereby enabling the construction of a homology model for MLH1 using the “FRankenstein's Monster” approach [56, 57]. That structural model was used to analyze 19 alterations connected to Lynch syndrome and to identify three alterations that decrease the efficiency of MMR in human by interfering with the MLH1-PMS2 dimerization, confirming that they are pathogenic, and suggesting that defective dimerization underlies their deleterious effect [50].

### 3.2. Methods for Predicting Protein-DNA Interactions

When analyzing enzymes acting on DNA, it is often important to know which parts of them interact with the substrate. Prediction of DNA-binding residues is facilitated by the knowledge of protein structure, either from experiment or from prediction (see above). An example of a bioinformatics online tool for structure-based prediction of DNA-binding residues is “*DISPLAR*” (http://pipe.scs.fsu.edu/displar.html), which uses a machine learning approach [58]. There are also methods, available as web services, enabling prediction of DNA-binding from protein sequence alone. Examples include “*BindN*+” (http://bioinfo.ggc.org/bindn+/) [59], “*DISIS*” (http://www.predictprotein.org/) [60], and “*DNABindR*” (http://turing.cs.iastate.edu/PredDNA/predict.html) [61]. 

If 3D structures of the components are known, it is also possible to obtain a three-dimensional model of protein-DNA complexes. The “*HADDOCK*” server (http://haddock.chem.uu.nl/) uses a flexible docking approach to build a complex from two or more separate protein and DNA structures [62]. It takes into account additional information such as distances between interacting residues and includes them as “ambiguous interaction restraints”. This allows to use results from experimental analyses like mutation, crosslinking, and footprinting experiments or computational predictions made, for example, by the above-mentioned bioinformatics methods. It is important to note that HADDOCK generates a complex structure for all given components, but it does not evaluate whether the given components really interact and does not enable the modeling of large conformational changes. Also, identifying the correct interaction region is the most error-prone step, which is why accurate experimental knowledge is essential to obtain reliable structures. The HADDOCK developers also provide an extensive dataset of protein-DNA complexes that can be used for benchmarking purposes [63]. An alternative approach is to build models with other methods, without the use of experimental data, and then use the “*FILTREST3D*” method developed in the laboratory of the authors [64] to rank them according to the extent of agreement with the restraints.

### 3.3. Methods for Predicting the Effects of Amino Acid Substitutions

As illustrated by the example of the MLH1 protein, prediction of mutation/substitution effects on protein structure and function, and linking them to the relevant phenotype can be very useful in the study of DNA repair proteins. “*SNPs3D*” (http://www.snps3d.org/) [65] is an online tool that returns predictions of functional effects of nonsynonymous SNPs stored in the NCBI dbSNP database; currently it does not make predictions for altered sequences submitted by the users. There are a few predictive online methods that use protein structure (solved experimentally or modeled) to infer the effect of user-defined amino acid substitutions. “*CUPSAT*” (http://cupsat.tu-bs.de/) (Cologne University Protein Stability Analysis Tool) [66] predicts Gibbs-free energy changes associated with amino acid substitutions, based on analyzing of residue interactions with its 3D environment. “*PopMusic*” (http://babylone.ulb.ac.be/popmusic/) [67] evaluates the changes of protein stability resulting from single-residue or multiple substitutions. “*I-Mutant 2.0*” (http://gpcr2.biocomp.unibo.it/cgi/predictors/I-Mutant2.0/I-Mutant2.0.cgi) [68] also predicts protein stability changes upon single-site substitutions. It can be used both as a classifier for predicting the sign of the protein stability change upon mutation and as a regression estimator for predicting the related Gibbs-free energy changes. “*MUpro*” (http://www.ics.uci.edu/~baldig/mutation.html) [69] is a set of machine learning programs to predict how single-site amino acid substitutions affect protein stability. The server accepts single protein sequences or sequences with a predicted tertiary structure of the protein as an input.

There are also methods that predict mutation/substitution effects based on sequence information alone. “*PolyPhen*” (Polymorphism Phenotyping) (http://genetics.bwh.harvard.edu/pph/) [70] predicts the possible impact of an amino acid substitution on the structure and function of human proteins, based on straightforward empirical rules. “*SIFT*” (http://sift.jcvi.org/) [71] predicts whether an amino acid substitution (AAS) affects protein function based on analysis of sequence profiles. It can be applied to study naturally occurring nonsynonymous polymorphisms as well as laboratory-induced missense mutations. “*MutPred*” (http://mutpred.mutdb.org/) [72] is a web application that predicts the gain/loss of 14 different structural and functional properties (for instance, gain of helical propensity or loss of a phosphorylation site). It also classifies an amino acid substitution as disease-associated or neutral in human. “*PhD-SNP*” (http://snps.uib.es/phd-snp/PhD-SNP.html) [73] is another machine-learning method for predicting whether a phenotype derived from a nonsynonymous SNP could be related to a genetic disease in humans. It is optimized to predict if a given point mutation can be classified as a disease-related or a neutral polymorphism.

### 3.4. Predicting Cancer Outcome

A tool which facilitates the analyses of cancer-related proteins, genes and pathways is CAERUS [39]—a tool for predicting cancer outcomes using relationships between protein structural information, protein networks, gene expression data, and mutation data (http://www.oicr.on.ca/research/ouellette/caerus/). This tool was developed in order to identify a list of gene signatures and to better predict cancer by investigating the changes in gene expression profiles caused by disruptions between protein-protein interactions and domain-domain interactions in the human interactome. As the authors of CAERUS indicate, it was tested on a set of well-documented breast cancer patients, which suggests that the disrupted interactome is important to determine patient prognosis. They also declare that this approach is robust if tested on other independent data sets and therefore offers a promising prognostic tool to classify different cancer outcomes. As DNA repair is closely connected to cancer, this service can be used in the analysis of proteins and genes related to oncogenesis. 

## 4. Summary

DNA repair is currently covered by a few dedicated databases. While REPAIRtoire and repairGenes focus on this topic, information is also available via general-purpose pathway databases. The main bottlenecks are the data collection and standardization. For instance, there is no specialized, universal ontology and no standards to describe entities and processes involved in DNA repair. Connecting the known “parts” such as enzymes, to pathways and processes in a formalized way that at the same time provides more insight into DNA repair processes, is probably the biggest challenge for the bioinformatics of DNA repair in the nearest future. It may be necessary to extend the currently established GO ontology by a vocabulary that will allow for describing repair processes on the protein complex and reaction level. A particular challenge is to find a consistent and appealing way to represent repair processes visually, and to include not only 3D descriptions, but also the dimension of time. The development and application of new computer programs for simulating and visualizing molecular processes involving multiple components will certainly contribute to our understanding of the complex process of DNA repair. In particular, it may help in the identification of new biomarkers, in predicting the possible side-effects of drugs based on personal genome information, and in the development of new therapeutic agents to restore the proper function of DNA repair proteins affected by disease-causing mutations.

## Figures and Tables

**Table 1:** Databases dedicated to DNA repair and general-purpose databases relevant to DNA repair.

Name	url	Reference	Description
Databases dedicated to DNA repair			

REPAIRtoire	http://repairtoire.genesilico.pl/	[22]	Database of DNA repair pathways
repairGENES	http://www.repairgenes.org/	unpublished	Database of DNA repair genes
Human DNA Repair Genes	http://sciencepark.mdanderson.org/labs/wood/DNA_Repair_Genes.html	[17]	Database of human DNA repair genes
Repair-FunMap	currently unavailable	[23]	A database of interactions between proteins involved in DNA repair and other proteins

Other databases relevant to DNA repair			

KEGG	http://www.genome.jp/kegg/	[21]	Kyoto Encyclopedia of Genes and Genomes
Reactome	http://www.reactome.org/ReactomeGWT/entrypoint.html	[24]	Database of human pathways and reactions
GeneSNPs	http://www.genome.utah.edu/genesnps/		This Environmental Genome Project web resource integrates gene, sequence, and polymorphism data into individually annotated gene models. The human genes included are related to DNA repair, cell cycle control, cell signaling, cell division, homeostasis, and metabolism
Mouse Mutation Database	http://pathcuric1.swmed.edu/research/research.htm	[25]	The Database of mouse strains carrying targeted mutations in genes affecting cellular responses to DNA damage
BioCyc (EcoCyc, MetaCyc)	http://biocyc.org/	[26]	Experimentally studied metabolic pathways and enzymes from more than 1,500 organisms
BRENDA	http://www.brenda-enzymes.org/	[27]	The main collection of enzyme functional data
Pathway Commons	http://www.pathwaycommons.org/pc/	[28]	A collection of publicly available pathway data from multiple organisms
NGSethDB	http://bioinfo2.ugr.es/NGSmethDB/gbrowse/hg19/	[29]	Database for next-generation sequencing single-cytosine-resolution DNA methylation data
DNAreplication	http://DNAreplication.net/	[30]	Database for the eukaryotic DNA replication community
MethyCancer	http://methycancer.psych.ac.cn/	[31]	Links between DNA methylation levels and cancer
PubMeth	http://matrix.ugent.be/pubmeth/	[32]	Links between DNA methylation levels and cancer
MethDB (2009)	http://www.methdb.de/	[33]	The database for DNA methylation and environmental epigenetic effects
OriDB	http://www.oridb.org/index.php	[34]	Confirmed and predicted DNA replication origin sites
REBASE	http://rebase.neb.com/rebase/rebase.html	[35]	Enzymes and genes for DNA restriction and modification in prokaryotes
ROSPath	http://rospath.ewha.ac.kr/	[36]	Reactive oxygen species (ROS) signaling pathway proteins
Pathguide	http://www.pathguide.org/	[37]	A listing of pathway, signal transduction, and protein-protein interaction databases
CREMOFAC	http://www.jncasr.ac.in/cremofac/	[38]	Chromatin remodeling factors
DAnCER	http://wodaklab.org/dancer/	[39]	Disease-Annotated Chromatin Epigenetics Resource
Telomerase database	http://telomerase.asu.edu/	[40]	Sequences and structures of the RNA and protein subunits of telomerase, mutations of telomerase components
Replication Domain	http://www.replicationdomain.com/	[41]	Replication timing database and genome-wide data visualization tool
